RETRACTED

# Downregulation of *MDR1* Gene by Cepharanthine Hydrochloride Is Related to the Activation of c-Jun/JNK in K562/ADR Cells

**DOI:** 10.1155/2014/164391

**Published:** 2014-10-16

**Authors:** Li Han, Yafeng Wang, Xiaojuan Guo, Yubing Zhou, Jingmin Zhang, Ning Wang, Jinhua Jiang, Fang Ma, Qingduan Wang

**Affiliations:** ^1^Zhang Zhongjing College of Chinese Medicine, Nanyang Institute of Technology, China; ^2^School of Pharmaceutical Sciences, Zhengzhou University, China; ^3^Department of Pharmacy, First Affiliated Hospital of Zhengzhou University, China; ^4^Henan Academy of Medical and Pharmaceutical Sciences, Zhengzhou University, Zhengzhou Henan 450052, China

## Abstract

The purpose of the study was to determine the signal transduction mechanism of cepharanthine hydrochloride (CH) on reversing tumor multidrug resistance. RT-PCR and Western blot analysis were used to determine the effects of CH on the expression of *MDR1* mRNA and P-glycoprotein in K562/ADR cells when CH was used alone and combined with SP600125, a JNK inhibitor, to explore the effects of CH on JNK pathway. Western blot analysis was used to determine the effects of CH on c-Jun protein expression and phosphorylation, to explore the regulating effects of CH on c-Jun and phosphorylated c-Jun (p-c-Jun) proteins. Our results showed that the inhibitory effect of CH on* MDR1* mRNA increased with the concentrations of CH (5.0, 10.0, and 20.0 *μ*M) and the inhibitory effects of CH on *MDR1* mRNA and P-glycoprotein increased with the incubation time of CH (0, 12, 24, 36, and 48 hours). The inhibitory effect was weakened after CH combined with SP600125. The expressions of c-Jun and p-c-Jun proteins increased with the incubation time of CH (0, 6, 12, and 24 hours). These findings suggest that CH downregulated the expressions of *MDR1* mRNA and P-glycoprotein in a time and concentration manner; the mechanism may be mediated via activating c-Jun/JNK pathway.

## 1. Introduction

Chemotherapy is one of the main treatment strategies for cancer patients currently. However, it is more and more serious that the multidrug resistance (MDR) occurred in the cancer patients as the anticancer drugs are widely used, which affected the patients' treatment directly. The overexpression of P-glycoprotein (P-gp), encoded by multidrug resistance gene* MDR1*, is one of the important mechanisms involved in MDR [1–3]. For that reason, it is a problem that should be solved quickly to search for MDR reversor and improve the chemotherapy sensitivity for medicine academia currently.

Natural source compounds have become the new trend of discovering the fourth-generation P-gp inhibitors because they are less toxic and more potent than the disappointing previous MDR modulators [4–6]. Cepharanthine hydrochloride (Figure 1), manufactured by salification from cepharanthine (CEP), which is a biscoclaurine alkaloid, extracted from* Stephania cepharantha Hayata*, has a reversed effect involved in multimechanisms from our previous studies [7–9]. In recent years, it is reported that CH has MDR-reversing effect and one of the reversing mechanisms is to inhibit the P-gp expression and function in MDR cancer cells [10, 11].

RETRACTED

Mitogen-activated protein kinase (MAPK) family has a vital role to play in regulating gene expression. c-Jun NH_2_-terminal kinase (JNK) is one of the members of MAPK family. Growing evidence suggests that JNK is closely related to the occurrence of MDR [12–14]. The signals relayed by JNK through c-Jun regulate a range of cellular processes including cell proliferation, tumorigenesis, apoptosis, and embryonic development.* MDR1* gene is also regulated through c-Jun in transcriptional level [15, 16]. Therefore, a new possible therapeutic target of reversing MDR and improving the effectiveness of chemotherapy is to regulate JNK pathway.

To the best of our knowledge, it remains unclear whether JNK associates with the regulation and expression of P-gp by CH on reversing MDR. The purpose of the study is to determine the signal transduction mechanism of CH on reversing MDR in the human chronic myeloid leukemia Adriamycin-tolerance K562/ADR cell line.

## 2. Methods

### 2.1. Reagents

CH was provided by Henan Academy of Medical and Pharmaceutical Sciences (Zhengzhou, Henan, China). SP600125 was purchased from Sigma-Aldrich (St. Louis, MO, USA). RPMI-1640 was purchased from Life Technologies (Grand Island, NY, USA). Anti-P-gp, c-Jun, p-c-Jun, and anti-*β*-actin primary and horseradish peroxidase (HRP)-conjugated secondary antibodies were purchased from Santa Cruz Biotechnology (Santa Cruz, CA, USA). ECL detection kit was purchased from Beyotime Institute of Biotechnology (Jiangsu, China).

### 2.2. Cell Lines and Cell Culture

K562 cells and K562/ADR cells were purchased from Shanghai Institutes for Biological Sciences, Chinese Academy of Sciences (Shanghai, China). The two cell lines were cultured in RPMI-1640 culture medium with 10% fetal bovine serum (FBS) at 37°C in a humidified atmosphere of 5% CO_2_. When the cells reached confluency, they were harvested and plated for either subsequent passages or drug treatments. The trypan blue exclusion test was used throughout the experiments to check cell viability.

### 2.3. Cell Growth Inhibition Assay

Chemosensitivity* in vitro* was measured by MTT assay. Briefly, the cells were harvested in exponential growth and seeded into 96 well plates at a density of 2.0 × 10^4^ cells per well in a final volume of 180 *μ*L with or without 5 *μ*M of CH or VER. After a 48 h incubation, 20 *μ*L of MTT was added to each well and further incubated for 4 h. The resulting formazan was dissolved with 200 *μ*L of dimethyl sulfoxide after aspiration of the culture medium. The plates were shaken for 5 min with a plate shaker and the absorbance was measured at 570 nm using a Bio-Rad ELISA plate reader (Bio-Rad, CA, USA). The fractional absorbance was calculated by the following formula: % cell survival = (mean absorbance in test well)/(mean absorbance in control wells) × 100%. IC_50_ was calculated from the cytotoxicity curves. The degree of resistance was calculated by dividing the IC_50_ for the MDR cells by that for the parental sensitive cells. The reversal fold of MDR was calculated by dividing the IC_50_ for cells to the anticancer drug in the absence of the modulator by that in the presence of the modulator.

RETRACTED

### 2.4. RT-PCR Analysis

To study the effects of CH on* MDR1* mRNA expression, the K562/ADR cells at a density of 1 × 10^5^/mL in exponential growth were exposed to 5.0, 10.0, and 20.0 *μ*M of CH for 48 h or were exposed to 10.0 *μ*M of CH for 12, 24, 36, and 48 h. For the investigation of the effects of CH on JNK signal transduction pathway in mRNA level, the K562/ADR cells were treated with 10.0 *μ*M of CH or 2.0 *μ*M of SP600125 along or CH plus SP600125 for 48 h. The total RNA isolation was performed with TRIZOL (Invitrogen, USA). All RNA preparation and handling steps took place in a laminar flow hood, under RNAse-free conditions. The isolated RNA from each fraction was dissolved in 20 *μ*L of RNAse-free water and stored at −80°C until used. cDNA synthesis was performed at 37°C for 15 min and 85°C for 5 sec using the Primer Script RT reagent Kit (TaKaRa Biotechnology, Dalian, China) in a total volume of 20 *μ*L according to the manufacturer's instructions. The primers sequences used for amplification of* MDR1* and* GAPDH* were shown in Table 1. The PCR cycling conditions comprised a denaturation step for 5 min at 95°C, followed by 35 cycles of denaturation (94°C for 15 s), annealing (58°C for* MDR1* and 57°C for* GAPDH* for 30 s), and extension (72°C for 30 s). After the last cycle, all PCR products were subjected to a final extension for 5 min at 72°C. PCR products were combined and then electrophoresed on 1.5% agarose gels containing ethidium bromide. Autoradiographic films of the RT-PCR assays were subjected to densitometric analyses using a KODAK Gel Logic 100 Image Station (Eastman Kodak, Rochester, NY, USA).

### 2.5. Western Blot Analysis

To study the effects of CH on c-Jun and phosphorylated c-Jun (p-c-Jun) expression, the K562/ADR cells were treated with 10.0 *μ*M of CH for 6, 12, and 24 h. For the investigation of the effects of CH on JNK signal transduction pathway in protein level, protein extracts for gel-electrophoresis were made from the cells treated as above according to standard techniques. Briefly, proteins were solubilized and then fractionated by sodium dodecyl sulfate polyacrylamide gel electrophoresis (SDS-PAGE). Western blotting analysis was performed by a slight modification of the method described previously [17]. Polyvinylidene fluoride membranes were incubated with primary antibodies (diluted 1 : 1,000): Pgp, p-c-Jun, c-Jun, and *β*-actin. The membranes were washed and incubated with HRP-conjugated secondary antibodies (diluted 1 : 2,000) for 1 h. The proteins were then detected using the ECL detection kit.

RETRACTED

### 2.6. Statistical Analysis

Data are the means ± SD from triplicate samples of at least three independent experiments. Differences between the mean values were analyzed by two-sample Student's *t*-test and one-way analysis of variance; the results were considered statistically significant when *P* < 0.05.

## 3. Results

### 3.1. Effect of CH on Reversing MDR* In Vitro*

The K562/ADR cells were approximately 31-fold resistant to ADR in comparison with the K562 cells. In drug-resistant K562/ADR cells, coincubation of CH with ADR resulted in a significant increase in the cytotoxicity of ADR; the IC_50_ dropped drastically from 13.97 ± 0.30 to 1.62 ± 0.10 *μ*M. While coincubation of the same concentration of VER resulted in a slight increase in the cytotoxicity of ADR, the IC_50_ shifted to 6.07 ± 0.18 *μ*M. However, this effect of CH or VER was not observed in parental K562 cells (Table 2).

### 3.2. Downregulation of* MDR1* mRNA and P-gp by CH

RT-PCR analysis showed that the level of* MDR1* mRNA decreased significantly after treatment with 10.0 *μ*M of CH (Figure 2(a)) and the level of* MDR1* mRNA partially decreased by 5.0 *μ*M of CH and completely by 20.0 *μ*M of CH in 48 h (Figure 2(b)), suggesting the downregulation of* MDR1* mRNA by CH in a time- and concentration-dependency. Western blot analysis showed that the level of P-gp decreased progressively from 24 to 48 h in a time-dependent manner after treatment with 10 *μ*M of CH (Figure 2(c)).

JNK activity is required for the downregulatory effect by CH on* MDR1* mRNA and P-gp.

We then examined whether the downregulation of P-glycoprotein by CH required JNK activity. After the cells were treated with 10.0 *μ*M of CH plus the JNK inhibitor SP600125 (2.0 *μ*M) for 48 h, the levels of* MDR1* mRNA and P-gp increased compared with that in the cells treated with 10.0 *μ*M of CH alone using RT-PCR and Western blot analysis (Figures 3 and 4), suggesting that SP600125 inhibited CH-induced downregulation of* MDR1* mRNA and P-gp expression in terms of both mRNA and protein level.

RETRACTED

### 3.3. CH Induces Activation of JNK in K562/ADR Cells

We sought to further confirm the above-mentioned findings by analyzing the transcription factor c-Jun and the substrate for JNK using Western blot. After treatment of the K562/ADR cells with 10.0 *μ*M of CH, c-Jun and phosphorylation-c-Jun (p-c-Jun) protein levels began to rise from 6 h (Figure 5), suggesting that CH increased both phosphorylation and expression of c-Jun in a time-dependent manner.

## 4. Discussion

MDR is complex biological processes that involve many MDR transporter proteins, genes, and signal transduction. Although researches have advanced greatly in MDR, it remains a formidable problem in clinical treatment. Statistics show that cancer deaths are on the rise all around the world and there will be more than over 11 million cancer deaths by 2020 [18]. More than 90% of all cancer deaths are considered to be associated with MDR [19]. A lot of researches currently are just focusing on a certain kind of resistance mechanisms designed to block the MDR, which may not be completely reversed. On the contrary, a research according to the different mechanisms simultaneously may be more effective to reverse the MDR.

In recent years, CH or CEP has been reported to induce apoptosis of human leukemia cell line and hematoma cell line [20], decrease the activation of GST-*π* and NF-*κ*B, and increase the activation of DNA Topo II to reverse MDR, suggesting that the reversing effect of CH involves multimechanisms. In recent years, the relationship between signal transduction pathway and MDR is becoming a hot research area gradually. Recent evidence indicates that pumping out xenosubstance is an important defense mechanism of the cell responding to stressful stimuli, while the regulation of* MDR1* expression often involves stress reaction and signal transduction [21], for example, JNK and NF-*κ*B. JNK is a stress-activated protein kinase that can be induced by inflammatory cytokines, bacterial endotoxin, osmotic shock, UV radiation, and so on. It has been reported that NF-*κ*B and JNK are functionally interconnected; activation of NF-*κ*B inhibits the activation of JNK and vice versa [22]. Our previous study has demonstrated that CH has weak antitumor effect [23]; other researchers reported that the effect was related to inhibiting the activation of NF-*κ*B [24]. In the meanwhile, the NF-*κ*B inhibition effect is one of the MDR reversing mechanisms of CH [11]. In view of this, we further investigated whether CH plays its P-gp inhibition effect is related to regulating the JNK pathway.

RETRACTED

SP600125, a reversible ATP-competitive inhibitor, specifically inhibits activation of the JNK in response to a variety of stress stimuli [25, 26]. In order to determine whether activation of JNK is directly associated with the P-gp expression in K562/ADR cells, we sought to block JNK activity using SP600125 and to determine the effect on the extent of inhibiting P-gp expression induced by CH. Our results showed that both the* MDR1* mRNA and P-gp expression increased after CH co-incubated with SP600125 in K562/ADR cells, suggesting CH induced* MDR1* mRNA and P-gp expression down-regulation is implicated in activating JNK. c-Jun is a protein that forms the activator protein 1 (AP-1) early response transcription factor. It is well known that c-Jun can be activated through double phosphorylation on serine 63 and 73 by the JNK pathway but has also a phosphorylation-independent function [27, 28]. The data presented here showed that CH promoted c-Jun expression and phosphorylation in K562/ADR cells in a time dependence manner, suggesting that c-Jun may be play an important role in downregulation of* MDR1* and P-gp expression.

It is worthwhile to note that the role of JNK pathway in the development of MDR is debated. Sui et al. [29] reported that inhibition of JNK downregulates the expression of* MDR1*/P-gp in resistant HCT8/V cells. While our results are in line with those in the papers by Zhou et al. [13], Miao and Ding [15], that is, the activation of JNK is related to the downregulation of* MDR1*/P-gp expression. This may reflect a complicated nature of* MDR1*/P-gp regulation by JNK with the involvement of P-gp modulators.

In conclusion, these results for the first time demonstrate that CH downregulates* MDR1* mRNA and P-gp expression by activating JNK/c-Jun. However, other signaling molecules may be also involved in the regulation of the activity of JNK in K562/ADR cells. Further studies are needed to explore how JNK and other signaling molecules interact in the regulation of P-gp-mediated MDR by CH in MDR cells.

## Figures and Tables

**Figure 1:** The chemical structure of CH used in the present study.

**Figure 2:** Effects of CH on* MDR1* mRNA and P-gp expression in K562/ADR cells. RT-PCR and Western blot analyses were performed to analyze* MDR1* mRNA and P-gp expression in K562/ADR cells. Time dependency ((a) and (c)) and concentration dependency (b) of* MDR1* mRNA and P-gp expression in 48 h after incubation with CH were examined.

**Figure 3:** Effects of the JNK inhibitor SP600125 on CH-induced downregulation of* MDR1* mRNA expression by RT-PCR analysis in K562/ADR cells (1 × 10^6^). CH-induced downregulation of* MDR1* mRNA expression was abolished partly when combined with SP600125 (2.0 *μ*M).

RETRACTED

**Figure 4:** Effects of the JNK inhibitor SP600125 (2.0 *μ*M) on CH-induced downregulation of P-gp expression by Western blot analysis in K562/ADR cells (1 × 10^6^). CH-induced downregulation of P-gp expression was abolished partly when combined with SP600125 (2.0 *μ*M).

**Figure 5:** Effects of CH on c-Jun and phosphorylated c-Jun (p-c-Jun) expression by Western blot analysis in K562/ADR cells (1 × 10^6^). Time dependency of c-Jun and p-c-Jun expression after incubation with 10.0 *μ*M of CH was examined.

**Table 1:** Primers and annealing temperatures for *MDR1* and *GAPDH*.

	Forward	Reverse	Annealing temperatures	Predicted size in bp
*MDR1 *	5′-CTG CTT GAT GGC AAA GAA ATA AAG-3′	5′-GGC TGT TGT CTC CAT AGG CAA T-3′	58°C	130

*GAPDH *	GAG TCA ACG GAT TTG GTC GT	GAC AAG CTT CCC GTT CTC AG	57°C	196

**Table 2:** Cytotoxicity of ADR alone and in combination with VER or CH in K562 and K562/ADR cells *in vitro*.

Drug and concentration	IC_50_ (*μ*M)		Resistance times	Reversing times
	K562	K562/ADR		
ADR	0.45 ± 0.11	13.97 ± 0.30^*^	31.04	
ADR + CH (5 *μ*M)	0.44 ± 0.12	1.62 ± 0.10^∗△^	3.68	8.43
ADR + VER (5 *μ*M)	0.46 ± 0.07	6.07 ± 0.18^∗△☆^	13.19	2.35

Cells were exposed to various concentrations of ADR, with or without 5 *μ*M CH, or VER for 48 h. ∗*P* < 0.05 compared with K562 treated with ADR, or ADR cotreated with CH or VER, ^△^ *P* < 0.05 compared with K562/ADR treated with ADR, ^☆^ *P* < 0.05 compared with K562/ADR treated with ADR plus CH.
